# The Role of Pulmonary Function Test for Pulmonary Arterial Hypertension in Patients with Connective Tissue Disease

**DOI:** 10.1155/2022/6066291

**Published:** 2022-09-29

**Authors:** Jiangbiao Xiong, Jianbin Li, Yiping Huang, Fan Yang, Rui Wu

**Affiliations:** The First Affiliated Hospital of Nanchang University, Nanchang 330006, China

## Abstract

*Objective*: The study aimed to investigate the value of pulmonary function test (PFT) in evaluating and predicting pulmonary arterial hypertension (PAH) in patients with connective tissue disease (CTD). *Methods*: This was a prospective observational study recruiting patients diagnosed with CTD-PAH. Patients with interstitial lung disease and pulmonary hypertension induced by other causes were not eligible for enrollment. All patients were assessed for PAH every 1–3 months. A patient was considered to have clinical improvement if the grade of risk stratification declined or at least two parameters improved during follow-up, otherwise no improvement. *Results*: A total of 31 patients with CTD-PAH were recruited in this study. Nearly 70% of patients had declined forced vital capacity (FVC), 60% had declined total lung capacity and maximum expiratory flow at 50% of vital capacity, and 95% had normal or mild decline in forced expiratory volume in 1 second (FEV1)/FVC. A decline in diffusing capacity of the lung for carbon monoxide (DLCO) was present in 96% of patients, and 60% were moderate to severe. Furthermore, 50% of patients had an FVC/DLCO ratio of less than 1.4. Univariate analysis showed that FEV1/FVC, DLCO, and FVC/DLCO were associated with disease prognosis. After adjusting for age as a confounding factor, multivariate logistic regression analysis revealed that DLCO was an independent predictive factor for the prognosis of CTD-PAH. *Conclusion*: The pulmonary function of patients with CTD-PAH is abnormal in parameters such as lung volume, small airway, and gas exchange. PFT can reveal complex pathophysiological changes in the lungs of CTD-PAH patients and predict prognosis.

## 1. Introduction

Pulmonary hypertension (PH) refers to a pathophysiological syndrome of right heart failure caused by a variety of etiologies that cause pulmonary vascular bed involvement to progressively increase pulmonary circulatory resistance [1]. Among many causes of PH, connective tissue disease-associated pulmonary arterial hypertension (CTD-PAH) accounts for about 25% [2]. PAH is one of the serious complications of CTDs [3]. Compared with idiopathic pulmonary arterial hypertension (IPAH), patients with CTD-PAH have a worse prognosis [4]. Early identification, regular assessment, and targeted treatment are important strategies to improve the prognosis of PAH [5, 6]. Right heart catheterization (RHC) is the gold standard for the diagnosis of PAH, but it is not suitable for the screening and evaluation of PAH because of its invasiveness and complicated operation [7]. Echocardiography is usually used clinically as the primary screening method for PAH, but there are certain differences compared with the results of RHC [8–11]. In PAH, pulmonary vascular endothelial proliferation, thickening of the vascular wall, and reduction of pulmonary vascular bed can lead to a decrease in diffusing capacity of the lung for carbon monoxide (DLCO), and the decline in DLCO is related to the severity of PAH [12, 13]. It is generally believed that PAH does not have ventilatory disorders [14]. Therefore, pulmonary function test (PFT) is recommended as a simple and easy auxiliary screening method for PAH [15]. However, some studies have found that peripheral small airway obstruction is common in all types of PH, including CTD-PAH [16–18]. The higher the World Health Organization functional class (WHO FC), the more serious the peripheral small airway obstruction [18]. In addition, there are studies showing that PAH has restrictive ventilation difficulties [19]. Although many studies believe that the decline of DLCO can be used as a clue for screening PAH, Mukerjee, George, and Knight believe that DLCO lacks sensitivity and specificity in systemic sclerosis (SSc)-associated PAH [20]. This study aimed to investigate the value of PFT in evaluating and predicting CTD-PAH.

## 2. Materials and Methods

### 2.1. Subjects and Study Design

This was a prospective observational study recruiting patients diagnosed with CTD-PAH at the First Affiliated Hospital of Nanchang University from January 2021 to July 2021. All enrolled patients met international diagnostic or classification criteria for different types of CTD [21, 22]. The diagnostic criteria for PAH were as follows: mean pulmonary arterial pressure (mPAP) >20 mmHg, pulmonary artery wedge pressure (PAWP) <15 mmHg, pulmonary vascular resistance (PVR) > 3 Wood units, measured by RHC, or systolic pulmonary arterial pressure (sPAP) ≥40 mmHg by transthoracic echocardiography [23]. Patients with interstitial lung disease (ILD) and PH induced by other causes, such as IPAH, congenital heart disease, chronic obstructive pulmonary disease, and pulmonary thromboembolism, were not eligible for enrollment. The study conformed to the principles of the Declaration of Helsinki and was approved by the Ethics Committee of the First Affiliated Hospital of Nanchang University. Written informed consent was obtained from all individual participants.

All patients were assessed for PAH every 1–3 months by including N-terminal prohormone of brain natriuretic peptide (NT-proBNP), PFT, echocardiography, 6-minute walking distance (6MWD), WHO FC, and risk stratification according to the 2015 European Society of Cardiology (ESC)/European Respiratory Society (ERS) Guidelines for the diagnosis and treatment of PH [24] and were followed up for 6 months. A patient was considered to have clinical improvement if the grade of risk stratification declined or at least two parameters improved during follow-up, otherwise no improvement.

### 2.2. PFT

The MasterScreen PFT System (Jaeger, Baglia, Germany) was used to measure the pulmonary function of patients. Parameters including forced vital capacity (FVC), forced expiratory volume in 1 second (FEV1), maximum expiratory flow at 50% of vital capacity (MEF50), total lung capacity (TLC), and DLCO were tested. The data were expressed as the percentage of the measured value to the predicted value, and the percentage <80% was considered abnormal.

### 2.3. Statistical Analysis

For statistical analysis, the SPSS version 22.0 (IBM, Armonk, NY, USA) and GraphPad Prism 9 (GraphPad Software, San Diego, CA, USA) were used. Continuous variables were expressed as the mean ± standard deviation for normally distributed data or the median [interquartile range (IQR)] for nonnormally distributed data. Categorical variables were described as a number and a percentage of the total. To compare the differences between two groups, we used the independent samples *t*-test or Mann–Whitney *U* test for continuous variables and the chi-square test or Fisher's exact test for categorical variables. A one-way analysis of variance (ANOVA) was employed to compare differences among three groups. Logistic regression analysis was used to analyze the predictive value of pulmonary function parameters for the prognosis of CTD-PAH. All statistical tests were two-tailed, and *p* value < 0.05 was considered statistically significant.

## 3. Results

### 3.1. Baseline Characteristics

A total of 31 patients with CTD-PAH, including 22 patients with systemic lupus erythematosus (SLE) and 9 patients with systemic sclerosis (SSc), were recruited in this study. All patients were treated with PAH target therapy. Only 3 patients at low risk were treated with monotherapy, and the rest were treated with combination therapy. The baseline clinical characteristics were shown in Table 1.

As shown in Figure 1, nearly 70% of patients had declined FVC, 60% had declined TLC and MEF50, and 95% had a normal or mild decline in FEV1/FVC. A decline in DLCO was present in 96% of patients, and 60% were moderate to severe. Furthermore, 50% of patients had an FVC/DLCO ratio of less than 1.4.

### 3.2. Comparisons of Pulmonary Function Parameters among Different Risk Groups

The ANOVA test indicated that FEV1/FVC, MEF50, DLCO, and FVC/DLCO were significantly different among low risk, intermediate risk, and high risk groups (Table 2). In particular, DLCO declined significantly with the rise of risk stratification of PAH, while FEV1/FVC and FVC/DLCO were also significantly different among different risk groups, but there was no declining trend. Multiple comparisons showed that there was no significant difference in MEF50 between the low and intermediate risk groups, but there was a significant decline in the high risk group compared with the lower risk group.

### 3.3. Predictive Value of Pulmonary Function Parameters

After 6 months of follow-up in all patients, 17 patients were clinically improved and 14 were not. Univariate analysis showed that FEV1/FVC, DLCO, and FVC/DLCO were associated with disease prognosis (Table 3). After adjusting for age as a confounding factor, multivariate logistic regression analysis revealed that DLCO was an independent predictive factor for the prognosis of CTD-PAH [odds ratio (OR) 4.813, 95% confidence interval (CI) 1.039–22.300] (Table 4).

## 4. Discussion

CTD-PAH belongs to group I of PH, and its pathophysiological changes are pulmonary vascular endothelial dysfunction, vascular remodeling, and progressive occlusion of small pulmonary arteries <200 *μ*m in diameter [25, 26]. PFT can reflect the information of various physiological and pathological changes of the lung, including the ventilation function of the airway and the gas exchange function of the vascular interstitium [18]. The relationship between group I of PH and parameters related to pulmonary ventilation function is still controversial, but the decline of DLCO, a parameter reflecting gas exchange function, is considered to be a characteristic change of pulmonary function in most patients with PAH [27, 28]. The decline in DLCO is the comprehensive result of endothelial cell proliferation leading to thickening of alveolar capillary membranes, increased PVR leading to decreased pulmonary vascular blood volume, decreased right ventricular output, and local thrombosis [29]. In this study, 96% of patients with CTD-PAH had a decline in DLCO, and 60% of patients had a DLCO below 60%. Moreover, DLCO declined with rising risk stratification. Importantly, multivariate analysis found that DLCO was an independent predictive factor for the prognosis of CTD-PAH.

Studies have shown that TLC in 20–50% of patients with IPAH decline, but some studies have not found it [30]. This study indicated that 60% of CTD-PAH patients had declined FVC and TLC. The reason for lung volume limitation in patients with PAH remains unclear. One explanation is that pulmonary vascular enlargement may have a direct physical effect on the airway, limiting tracheal dilation by mechanical pressure on the airway [31]. In addition to the factors of enlarged pulmonary vessels, the subsequent enlargement of the atria and ventricles may lead to the displacement of lung tissue within the thoracic cavity and affect the lung volume [32]. Most studies show that FEV1/FVC is normal in group I of PH [33]. This study showed that 95% of patients with CTD-PAH had an FEV1/FVC above 70%. Nevertheless, it is not sufficient to conclude that there is no airway obstruction in PAH, because FEV1 does not change much when small airways are obstructed, and extensive small airway obstruction only causes a small decline in FEV1. This study showed that MEF50, a sensitive marker of small airway, declined in 60% of patients with CTD-PAH, of which 42% had a MEF50 below 60%. Moreover, the MEF50 in the high risk group was significantly lower than that in the low risk group, while there was no significant difference between the low and intermediate risk groups, suggesting that small airway obstruction was more common in CTD-PAH patients with high risk stratification [34]. As with lung volume, the cause of obstruction of the small airways in patients with PAH is also unclear. A possible histological explanation is that pulmonary artery thickening invades the adjacent airways, impairing airflow and causing airway obstruction [31, 32]. Some studies have also suggested that inflammatory cytokines in lung tissue not only play a role in pulmonary vascular remodeling but may also overflow from vessels to the airways, resulting in airway inflammation [35, 36]. Some substances that play a key role in the pathogenesis of PH, such as endothelin-1 and nitric oxide, can also affect the contraction and dilation of bronchi in vivo and vitro [37, 38]. We also observed improvement in TLC and FEV1/FVC after treatment of PAH, suggesting that the decrease in TLC and FEV1/FVC were related to PAH.

Some studies suggest that patients with PAH can have a mild decrease in FVC, but the decline in DLCO should be more significant [18]. Meanwhile, FVC and DLCO decreased synchronously in patients with ILD. Therefore, it is recommended to use FVC/DLCO to differentiate PAH from ILD. When FVC/DLCO is less than 1.4, the possibility of ILD is high, and when it is greater than 2, the diagnosis of PAH should be taken into consideration [39]. There are also studies finding that FVC/DLCO greater than 1.9 has a sensitivity and specificity of 87.5% and 100% in predicting PAH [40]. However, the results of this study showed that the FVC/DLCO of more than half of the patients with CTD-PAH was below 1.4, and only 10% of the patients had a ratio above 1.9, suggesting that the value of FVC/DLCO as a predictor of PAH is limited.

The study has several limitations. First, different types of CTD have different mechanisms of PAH, resulting in no significant difference in FVC/DLCO in this study. Second, only two types of CTD-PAH were included, which may lead to biased results. Third, the sample size was not large enough. A large-scale and multicenter study is needed in the future.

## 5. Conclusion

The pulmonary function of patients with CTD-PAH is abnormal in parameters such as lung volume, small airway, and gas exchange. PFT can reveal complex pathophysiological changes in the lungs of CTD-PAH patients and predict prognosis. Exploring the mechanism of abnormal pulmonary function may provide new directions for the treatment of CTD-PAH.

## Figures and Tables

**Figure 1:** Pie chart of different pulmonary function parameters. FVC: forced vital capacity; FEV1: forced expiratory volume in 1 second; MEF50: maximum expiratory flow at 50% of vital capacity; TLC: total lung capacity; DLCO: diffusing capacity of the lung for carbon monoxide.

**Table 1:** Baseline clinical characteristics of patients with CTD-PAH.

Characteristics	Value
Total number	31
SLE	22 (76.3%)
SSc	9 (23.7%)
Age (years)	42.32 ± 13.82
Female	30 (96.8%)
NT-proBNP (ng/L)	966.16 ± 906.13
Stabilization of CTD	21 (67.7%)
sPAP (mmHg)	47.84 ± 9.56
RAA (cm^2^)	18.52 ± 2.51
RVBD (cm)	3.59 ± 1.42
RAP (mmHg)	9.03 ± 3.69
TAPSE (mm)	16.17 ± 3.24
6MWD (m)	381.26 ± 69.42
WHO FC	
I	6 (19.4%)
II	13 (41.9%)
III	9 (29.0%)
IV	3 (9.7%)
Risk stratification	
Low risk	8 (25.8%)
Intermediate risk	15 (48.4%)
High risk	8 (25.8%)
FVC (%)	78.56 ± 15.76
FEV1/FVC (%)	83.00 ± 10.65
MEF50 (%)	70.27 ± 31.29
TLC (%)	80.97 ± 13.44
DLCO (%)	56.84 ± 17.39
FVC/DLCO	1.52 ± 0.72

SLE: systemic lupus erythematosus; SSc: systemic sclerosis; CTD: connective tissue disease; NT-proBNP: N-terminal prohormone of brain natriuretic peptide; sPAP: systolic pulmonary arterial pressure; RAA: right atrial area; RVBD: right ventricular basal diameter; RAP: right atrial pressure; TAPSE: tricuspid annular plane systolic excursion; 6MWD: 6-minute walking distance; WHO FC: World Health Organization functional class; FVC: forced vital capacity; FEV1: forced expiratory volume in 1 second; MEF50: maximum expiratory flow at 50% of vital capacity; TLC: total lung capacity; DLCO: diffusing capacity of the lung for carbon monoxide.

**Table 2:** Comparisons of pulmonary function parameters among different risk groups.

Parameters	Low risk	Intermediate risk	High risk	*P* value
FVC (%)	81.23 ± 15.20	76.80 ± 12.57	67.09 ± 22.31	0.104
FEV1/FVC (%)	85.03 ± 15.54	93.17 ± 8.65	83.03 ± 7.43	**0.029**
MEF50 (%)	69.88 ± 39.40	71.12 ± 26.32	35.81 ± 22.93	**0.021**
TLC (%)	82.25 ± 10.44	78.58 ± 11.29	74.59 ± 15.08	0.287
DLCO (%)	69.67 ± 7.62	48.89 ± 13.22	44.65 ± 16.44	**<0.001**
FVC/DLCO	1.18 ± 0.29	1.71 ± 0.74	1.52 ± 0.18	**0.014**

Bold values are statistically significant (*P* < 0.05). FVC: forced vital capacity; FEV1: forced expiratory volume in 1 second; MEF50: maximum expiratory flow at 50% of vital capacity; TLC: total lung capacity; DLCO: diffusing capacity of the lung for carbon monoxide.

**Table 3:** Comparisons of pulmonary function parameters between groups with and without improvement.

Parameters	Group without improvement (*n* = 14)	Group with improvement (*n* = 17)	*P* value
FVC (%)	74.21 ± 19.34	79.01 ± 11.85	0.558
FEV1/FVC (%)	90.09 ± 7.67	87.57 ± 14.80	**0.020**
MEF50 (%)	57.24 ± 30.81	71.64 ± 34.09	0.553
TLC (%)	75.03 ± 13.71	82.71 ± 8.54	0.058
DLCO (%)	43.13 ± 13.20	65.76 ± 9.47	**0.001**
FVC/DLCO	1.82 ± 0.72	1.22 ± 0.25	**0.002**

Bold values are statistically significant (*P* < 0.05). FVC: forced vital capacity; FEV1: forced expiratory volume in 1 second; MEF50: maximum expiratory flow at 50% of vital capacity; TLC: total lung capacity; DLCO: diffusing capacity of the lung for carbon monoxide.

**Table 4:** Logistic regression analysis for the predictive value of pulmonary function parameters.

Parameters	OR	95% CI	*P* value
TLC (%)	0.911	0.817–1.017	0.096
FEV1/FVC (%)	1.044	0.950–1.147	0.371
DLCO (%)	4.813	1.039–22.300	**0.045**

OR: odds ratio; 95% CI: 95% confidence interval. Bold values are statistically significant (*P* < 0.05). FVC: forced vital capacity; FEV1: forced expiratory volume in 1 second; DLCO: diffusing capacity of the lung for carbon monoxide.

## Data Availability

The data used to support the findings of this study will be available from the corresponding author upon reasonable request.
